RETRACTED

# Hypoxia‐Induced GST1 Exerts Protective Effects on Trophoblasts via Inhibiting Reactive Oxygen Species (ROS) Accumulation

**DOI:** 10.1155/2023/9391252

**Published:** 2023-01-25

**Authors:** Lingjuan Chen, Gaoli Chen, Lixuan Guo, Yaping Wang, Chengjin Ai

**Affiliations:** ^1^ Department of Laboratory Medicine, Hospital of Chengdu University of Traditional Chinese Medicine, Chengdu, 610072 Sichuan Province, China cdutcm.edu.cn; ^2^ Ophthalmology Department, Hospital of Chengdu University of Traditional Chinese Medicine, Chengdu, 610072 Sichuan, China cdutcm.edu.cn

## Abstract

Hypoxic conditions are a typical extrinsic factor for the modification of trophoblast biological functions, including cell proliferation, migration, and invasion. Hypoxia‐induced reactive oxygen species (ROS) accumulation causes chronic trophoblast injury and contributes to preeclampsia (PE). Glutathione‐S‐transferase P (GSTP1) is a main regulator of ROS. However, it is still unknown whether GSTP1 is involved in ROS regulation under hypoxic conditions. Here, we investigated the expression level of GSTP1 in first‐trimester villi placentas compared with full‐term placentas and the effect of hypoxic conditions on GSTP1. GSTP1 expression in first‐trimester villi placentas was much higher than that in full‐term placentas. After hypoxia exposure, GSTP1 was significantly upregulated in JEG3 cells, a trophoblast‐like cell line. Hypoxic‐induced GSTP1 scavenged ROS accumulated by hypoxia exposure, potentially by promoting GST activity. The inhibitory effects of hypoxia exposure on cell proliferation, migration, and invasion induced by hypoxia exposure were obviously reversed by overexpression of GSTP1. Hypoxia‐induced cell apoptosis was also reversed by GSTP1 overexpression, indicating the protective effects of GSTP1 against ROS‐induced cell injury. Moreover, overexpressed GSTP1 markedly promoted the cell proliferation, migration, invasion, and colony formation abilities in JEG3 cells, demonstrating that GSP1 also exerts promoting effects under normoxic conditions. These data show that hypoxia‐induced GSTP1 expression facilitates trophoblast cell proliferation, migration, and invasion and exerts protective effects under hypoxic conditions, which may play an important role during the increase in PE.

## 1. Introduction

Early in pregnancy, extra villous cytotrophoblast cells occlude the uterine spiral artery. In this progression, little maternal blood is observed in the intervillous space (IVS). However, at approximately 10–12 weeks of gestation, the maternal endothelial cells are replaced by cytotrophoblasts, and the spiral arterioles are remodeled to form large, low‐resistance blood vessels that transport more blood to the mother‐fetus interface [1]. Morphological modification in virtually all 100–150 spiral arteries in the placental bed is necessary for successful pregnancy [2]. Thus, before the tenth week of pregnancy, the placenta develops in a hypoxic environment, with oxygen levels of 2–3% O_2_ [3]. Changes in O_2_ tension in IVS play a physiological role in the differentiation and invasion of trophoblasts due to low levels of antioxidant enzymes in the placenta, which must be strictly controlled due to their association with pregnancy outcomes [4]. Genbacev et al. previously conducted in vitro studies and reported that hypoxia inhibited the invasion of primary trophoblast cells [5, 6]. Recently, studies in trophoblast‐like cell lines such as HTR‐8/SVNEO and JEG3 cells showed that genes related to cell migration and invasion were highly expressed [7], and in vitro cell migration and invasion capacities were upregulated under low‐O_2_ environments [8].

RETRACTED

Hypoxia is a pervasive irritant affecting a wide range of biological processes. Hypoxia induces the nuclear translocation and dimerization of oxygen‐labile *α*‐subunit (HIF*α*) and constitutively expressed *β*‐subunit (HIF*β*) to form HIFs (HIF1, HIF2, and HIF3), which then bind to the hypoxic response element of related genes [9]. Target genes are involved in glycolysis, erythropoiesis, and angiogenesis. Structural expression of HIF1*α* and HIF2*α* proteins in the human placenta, with peak mRNA and protein levels of HIF1*α* observed at 7–10 weeks gestation [10]; however, few studies have examined HIF3 expression in the placenta. Studies have shown that placentas from Arnt‐/‐, Hif1‐*α*‐/‐, or Hif2‐*α*‐/‐embryos show defects in defective trophoblast invasion and placental vascularization, leading to aberrant cell fate adoption [11]. It is also believed that chronic hypoxia is a main cause of placental diseases, including preeclampsia (PE) [12, 13]. Considering that trophoblast abnormalities are the main characteristic of PE, chronic hypoxia potentially results in placental diseases by inducing trophoblast injury.

Glutathione S‐transferases between glutathione (GSH) and lipophilic compounds neutralize toxic compounds, xenografts, and oxidative stress products. Protein kinase C alpha (PKC*α*) phosphorylation of GSTP1 serine has been reported to enhance GSTP1‐dependent cisplatin metabolism and human glioma cell resistance [13]. In addition, GST polymorphisms represent a risk factor for various cancers. For example, the GSTP1 gene Ile105Val polymorphism is involved in the development of glioma, prostate cancer, and other cancers [14, 15]. In addition, GSTP1 dimers are larger and cannot bind to the c‐Jun N‐terminal kinase (JNK) and inhibit its activation under conditions of reactive oxygen species (ROS) overexpression [16]. Notably, the GSTP1 inhibitor ezatiostat has been approved for evaluation in a Phase II clinical trial for the treatment of myelodysplastic syndrome, suggesting that GSTP1 inhibitors may be used in human cancers [17]. Since NADPH quinone oxidoreductase 1 (NQO1) and GSTP1 are Phase II detoxification enzymes that reduce quinone directly to hydroquinone and eliminate the formation of ROS from redox cycling [18], inhibition of NQO1 and GSTP1 may provide a potential solution for cancer treatment.

RETRACTED

The signal transducer and activator of transcription (STAT) family proteins are phosphorylated via Janus kinases (JAKs) in response to the binding of growth factors or cytokines to their corresponding receptors [19]. GSTP1 is reported to promote malignancies in colorectal cancer cells by activating STAT3 [20]. In this study, we aimed to investigate the effects of hypoxia stress on GSTP1 and its subsequent regulation of STAT3. We compared the expression levels of GSTP1 in villi and term placentas. After GSTP1 overexpression in trophoblast cells, its effects on proliferation, colony formation, and migration were evaluated. Then, the effects of hypoxia on GSTP1 and its subsequent protective effects were further measured. In addition, the regulatory effect of hypoxia‐induced GSTP1 on STAT3 was further analyzed.

## 2. Material and Methods

### 2.1. Sample Collection

The sample collection was performed as described previously [21]. Briefly, the first‐trimester chorionic villi samples (6, 6, 7, 7 weeks for each) were obtained and dissected out immediately after vacuum aspiration from women who underwent a legal termination of an apparently normal early pregnancy. Full‐term tissues (39, 39, 40, 40 weeks for each) were obtained from normal placenta after uncomplicated caesarean section deliveries. All samples were stored in liquid nitrogen for total protein extraction and fixed at 4°C using 4% paraformaldehyde for Immunohistochemistry (IHC). All samples were obtained from the Hospital of Chengdu University of Traditional Chinese Medicine. Experiment was approved by the Ethics Committees of Hospital of Chengdu University of Traditional Chinese Medicine.

### 2.2. Cell Culture and Transfection

Cells were seeded and cultured in an incubator at 37°C with 5% carbon dioxide/air atmosphere (21% O_2_, standard conditions). 24 hours later, the cells were maintained in an atmosphere of 21% O_2_ (normoxia group) or transferred to a tri‐gas incubator with 3% O_2_, 5% CO_2_, and 92% N_2_ (hypoxia group). For GSTP1 overexpression, lentivirus‐containing coding sequences of GSTP1 were bought from GeneCopoeia (Guangzhou, China) and were employed following standard protocols. Briefly, cells were seeded with 80% confluence, and lentivirus particles were added at multiplicity of infection (MOI) approximately 10 in the presence of 8 *μ*g/ml polybrene. Three days after transduction, 5 *μ*g/ml puromycin was added to medium to select for stably transduced cells. Medium was replaced for every two days until 90% of cells survived the selection without obvious cell damage.

RETRACTED

### 2.3. CCK‐8 Analysis

Cells were plated in 96‐well plates at a density of 5 × 10^3^ cells per well and maintained in complete medium supplemented with 10% heat‐inactivated (56°C, 30 min) fetal bovine serum (FBS, Gibco) and 1% antibiotics (penicillin/streptomycin, Gibco). 24 hours later,10 *μ*L of Cell Counting Kit‐8 (CCK‐8) solution were added to each well, after which the cells were incubated for 2 hours at 37°C. After incubation, absorbance was measured at 450 nm. The cell viability was measured every 24 hours from day 1 to 5.

### 2.4. Protein Extraction and Western Blotting

Cells were lysed and treated using SoniConvert® Tissue cell convertor (DocSense, Chengdu, China) by following manufacturer’s instructions in chilled lysis buffer containing 50 mM Tris‐HCl (pH 7.4), 150 mM NaCl, 1% Triton X‐100, 5 mM EDTA, 1 mM Na_3_VO_4_, 1 mM NaF, 10 *μ*M PMSF on ice for 10 min. The extracted protein concentration was measured using the BCA Protein Assay Kit (Thermo Scientific). For the western blot analysis, 20 *μ*g of protein extracts from each clone was loaded onto 10% sodium dodecyl sulfate‐polyacrylamide gel electrophoresis (SDS‐PAGE) gels and transferred to polyvinylidene difluoride membranes (PVDF, Roche Diagnostics). After blocking at room temperature for 1 hour, the protein was probed with primary antibodies, and an anti‐*β*‐actin antibody was used as a loading control. Signals were detected using an ECL chemiluminescence kit (Millipore Corporation, Billerica, MA, USA).

### 2.5. Immunohistochemistry

Fixed placental tissues were cut into 4 *μ*m thick sections. Dissected tissue slides were deparaffinized and rehydrated. Before blocking, the slides were pretreated with 3% hydrogen peroxide/methyl alcohol for 10 min to inhibit endogenous peroxidase activity. Non‐specific binding sites were blocked with 5% Bovine serum albumin (BSA) for 30 min at room temperature, and then the tissue sections were probed with primary antibody at dilution of 1 : 100 overnight at 4°C. The sections were then incubated with an HRP‐labeled anti‐rabbit/mouse IgG polymer (EnVision Detection Kit, Peroxidase/DAB, Rabbit/Mouse, Gene Tech, CA, USA) for 30 min at room temperature.

RETRACTED

### 2.6. Tumor Formation in Soft Agar

5 × 10^3^ cells were suspended in 0.35% biotechnology‐grade agarose (Bio‐Rad, Hercules, CA, USA) in complete medium and plated before solidifying on a solid 0.5% agarose with complete medium. Colonies were maintained for 14 days in a 37°C humidified incubator, after which they were stained with methylene blue (Sigma‐Aldrich, St. Louis, MO, USA) and counted.

### 2.7. Migration and Invasion

Migration was assessed in a Transwell chamber assay. Briefly, 1 × 10^4^ cells were seeded into cell culture inserts containing membranes with 8 *μ*m pores that were placed in wells containing cell culture medium with 2% FBS. 24 hours later, unmigrated cells were removed with cotton swabs, and migrated cells were fixed in cold methanol and stained with Diff‐Quick solution. Cells were imaged. Similar results were obtained in three independent experiments.

Invasion assay was performed using BD Transwell Invasion Chamber (BD Biosciences, Bedford, MA, USA). 1 × 10^4^ cells in complete medium with supplements described as before were added to the Matrigel chamber. Chambers were incubated overnight in a cell culture incubator, at 37°C, 5% CO_2_ atmosphere. 48 hours later, non‐invading cells were removed with a cotton swab. Invaded cells were sequentially transferred through a fixative, then 4% paraformaldehyde solution for 15 min at room temperature. After three washes using Phosphate‐buffered saline (PBS), invaded cells were allowed to air dry. Membranes were mounted onto slides using immersion oil and covered with a cover slip. Cells were counted using light microscopy at 40× magnification.

### 2.8. Apoptosis Analysis

Annexin‐V Apoptosis Detection Kit (Cell Signaling Technology) was used to quantify the levels of apoptosis according to the manufacturer’s instructions. Briefly, 1 × 10^6^ cells were trypsinized and collected by centrifugation at 4°C, 1000 *g* for 10 min. Then cells were incubated with Annexin V‐FITC and propidium iodide (PI). Apoptosis was analyzed by flow cytometry (Beckman, Navios) for the detection of Annexin V‐FITC. Data was analyzed using FlowJo. Experiments were performed at least three times, and statistical analysis was performed with GraphPad Prism.

### 2.9. GST Activity Assay

As previously reported [22], GST activity was analyzed by the increase of the absorbance at 340 nm at 25°C with reduced GSH and 1‐chloro‐2,4‐dinitrobenzene (CDNB) as substrates. The GST Assay Kit (Millipore Sigma, CS0410) was used per the manufacturer’s protocols. Briefly, 1 million cells were lysed in 50 *μ*L of sample buffer by sonication. Then 30 *μ*L of the samples were added into the assay cocktail (150 *μ*L of PBS at pH 6.5, 10 *μ*L of 100 mM CDNB, and 10 *μ*L of 100 mM GSH) in 96‐well plates and immediately analyzed in a plate reader. The change in absorbance (*Δ*A340) per minute, in the linear range of the plot, was calculated using equation (1):

(1) ΔA340min=A340340final read−Ainitial readreaction time min,

GST‐specific activity per million cells (*μ*mol/million/min) was calculated using equation (2):

(2) ΔA340/min×V mL×dilution/ε mM×Venz mL×density.

RETRACTED

For our assay using 96‐well plates, *ε* (mM) = 5.3 mM − 1; *V* (mL) = 0.2 mL; Venz (mL) = the volume of the enzyme sample tested; and density = number of cells used in cell lysate.

### 2.10. Statistical Analysis

Statistical analysis was conducted using one‐way ANOVA, and statistical significance was set at *p* < 0.05.

## 3. Results

### 3.1. GSTP1 Protein Levels Are High in First‐Trimester Villi

To explore the expression of GSTP1 in first‐trimester villi compared with normal full‐term placentas, we collected 4 first‐trimester chorionic villi samples (6, 6, 7, 7 weeks for each) and 4 full‐term placenta tissues (39, 39, 40, 40 weeks for each) and fixed immediately using paraformaldehyde. Then, samples were analyzed by performing IHC to localize GSTP1 protein expression in the human placenta, which demonstrate that GSTP1 was mainly expressed in cytoplasm of trophoblasts, and that trophoblast GSTP1 expression was obviously higher in first‐trimester villi than those in full‐term placentas (Figure 1(a)). Total protein extracted from these tissues were then fractionated by western blot and detected by immune blotting. Results also demonstrated that, in first‐trimester villi tissues, GSTP1 protein levels were obviously higher than those in full‐term placentas (Figure 1(b)). By considering that GSTP1 was mainly expressed in trophoblasts (Figure 1(a)), the difference in GSTP1 protein level is mainly due to those in trophoblasts.

Figure 1Detection of GSTP1 protein in first‐trimester villi and full‐term placenta tissues. (a) Placenta tissues collected from first‐trimester villi or full‐term patients were detected by performing ISH to evaluate the effects of GSTP1 protein. (b) Fresh placenta tissues were lysed and detected by performing western blot to detect GSTP1 protein levels.

**Figure:** (a)

**Figure:** (b)

### 3.2. JEG3 Cell Proliferation, Migration, and Invasion Are Promoted by Overexpressed GSTP1

To evaluate the exact role of GSTP1 in trophoblasts, in this study, trophoblast‐like cell line JEG3 was employed. After efficient introduction of GSTP1 into JEG3 (Figure 2(a)), cell viability was measured from day 1 to 5 after cells were seeded. As it is shown in Figure 2(b), introduction of GSTP1 significantly increased cell viability. Then, cell cycle phase distribution was measured by PI staining. As illustrated in Figure 2(c), overexpression of GSTP1 decreased proportion of G_1_/G_0_ phase and increased proportion of G_2_/M phase, which potentially results in increase in cell proliferation. We also detected colony formation, tumor formation, migration, and invasion after GSTP1 overexpression. Expectedly, it is observed that overexpressed GSTP1 increased colony formation (Figure 2(d)), tumor formation in soft agar (Figure 2(e)), migration (Figure 2(f)), and invasion (Figure 2(g)). These results indicate that overexpressed GSTP1 exerts critical roles in regulating both tumor‐like properties and trophoblast‐like properties in JEG3 cells.

RETRACTED

Figure 2Overexpression of GSTP1 promotes cell proliferation. (a) After GSTP1 overexpression by lentivirus infection, efficient overexpression of GSTP1 was detected by performing western blot. (b) After stable GSTP1 overexpression, cell viability was measured from day 1 to 5 by performing CCK‐8 assay, respectively. *P < 0.05, vs. vector group. (c) After being cultured for 24 hours on 6‐well plate, cells were collected and fixed by using 70% ethanol for 24 hours, and cell cycle distribution was measured by performing PI staining followed by flow cytometry analysis. *P < 0.05, vs. vector group. After GSTP1 overexpression stably, colony formation (d), tumor formation in soft agar (e), migration (f), and invasion (g) were analyzed. *P < 0.05, vs. vector group.

**Figure:** (a)

**Figure:** (b)

**Figure:** (c)

**Figure:** (d)

**Figure:** (e)

**Figure:** (f)

**Figure:** (g)

### 3.3. GSTP1 Expression Is Stimulated in JEG3 Cells Exposed to Hypoxia Condition (3% O_2_)

By considering that physiologically low levels of O_2_ are a critical factor involved in maintenance of normal pregnancy [5, 6], we then evaluated the effects of hypoxia condition (3% O_2_) on GSTP1 expression. After 12‐ or 24‐hour hypoxic incubation, HIF‐1a is obviously induced, indicating that hypoxic treatment was appropriately performed (Figure 3(a)) [25]. GSTP1 was also obviously stimulated after 12‐hour and 24‐hour hypoxic treatment, indicated that GSTP1 is a potential hypoxia‐sensitive gene (Figure 3(a)). After 24‐hour hypoxia treatment, ROS level is obviously increased, and introduction of GSTP1 obviously decreased hypoxic‐stimulated ROS (Figures 3(b) and 3(c)), which indicated that GSTP1 may inhibit ROS accumulation or promote ROS scavenge.

Figure 3GSTP1 is induced by hypoxia exposure and scavenged ROS. (a) After being culture in normoxia or hypoxia for 12 or 24 hours, western blot was performed to detect HIF‐1*α* and GSTP1 protein levels. (b) After being cultured under normoxia or hypoxia with overexpressed GSTP1, intracellular ROS was stained and imaged by using Olympus x71 microscope. (c) Accumulation of ROS was measured quantitatively. *P < 0.05, vs. normoxia group; ^#^ *P* < 0.05, vs. hypoxia/vector group.

RETRACTED

**Figure:** (a)

**Figure:** (b)

**Figure:** (c)

### 3.4. Overexpressed GSTP1 Is Critical for Inhibiting ROS Accumulation

GSTP1 is one of the glutathione‐S‐transferase (GST) family members that catalyze intracellular detoxification reactions by conjugating GSH [24]. Also, downregulation of GSTP1 or pharmacological inhibition of its activity increases ROS level [24]. By considering this, we further analyzed whether hypoxia‐induced GSTP1 stimulates its activity. After GSTP1 overexpression or hypoxia exposure, GST activity was promoted and was then inhibited by addition of GSTP1 inhibitor, TLK199 (Figure 4(a)). Moreover, after hypoxia exposure, ROS level was expectedly observed to be increased, which was further enhanced by addition of TLK199 (Figure 4(b)), which indicates that function GSTP1 is critical for scavenging ROS caused by oxidative stress.

Figure 4GSTP1 scavenged ROS accumulation. (a) After hypoxia exposure or TLK199 treatment, GST activity was measured quantitatively. *P < 0.05, vs. hypoxia group; ^#^ *P* < 0.05, vs. hypoxia/GSTP1 group. (b) ROS accumulation was measured. *P < 0.05, vs. hypoxia group; ^#^ *P* < 0.05, vs. hypoxia/GSTP1 group.

**Figure:** (a)

**Figure:** (b)

### 3.5. Overexpression of GSTP1 Reversed Cell Injury Caused by Hypoxia Exposure

By considering that ROS accumulation induced by hypoxia exposure is a main cause of cell injury, including decrease in cell viability and increase in ROS‐related apoptosis, we then evaluate the effects of overexpressed GSTP1 on all these behaviors. As it is illustrated in Figure 5(a), hypoxia treatment significantly decreased cell viability after 24‐hour exposure to hypoxia, and overexpression of GSTP1 significantly reversed the decrease in viability caused by hypoxia exposure. Expectedly, overexpression of GSTP1 also reversed the inhibitory effects of hypoxia exposure on migration and invasion (Figures 5(b) and 5(c)). By performing apoptosis analysis using Annexin V‐FITC/PI double staining followed by flow cytometry, hypoxia treatment for 48 hours significantly increased apoptosis (57.51 ± 2.56%), compared to normoxia group (7.46 ± 0.63%). Expectedly, overexpression of GSTP1 exerts protective effects on hypoxic‐induced apoptosis (22.57 ± 3.15%) (Figure 5(d)).

Figure 5Overexpressed GSTP1 exerts protective effects against hypoxia‐induced cell injury. (a) After being cultured under normoxia or hypoxia condition for 24 hours, cell viability was measured by performing CCK‐8 assay. *P < 0.05, vs. normoxia group; ^#^ *P* < 0.05, vs. hypoxia/vector group. After being cultured under normoxia or hypoxia condition for 24 hours, cell migration (b) and invasion (c) were detected, respectively. (d) After being cultured under normoxia or hypoxia condition for 48 hours, cells were collected and stained using Annexin V‐FITC/PI double staining, then stained cells were analyzed by performing flow cytometry assay. *P < 0.05, vs. normoxia group; ^#^ *P* < 0.05, vs. hypoxia/vector group.

RETRACTED

**Figure:** (a)

**Figure:** (b)

**Figure:** (c)

**Figure:** (d)

### 3.6. GSTP1 Induced Stimulated STAT3 Phosphorylation and Its Downstream Target Cyclin D1

STAT3, a critical transcriptional factor regulating tumorigenesis via modulating several activated oncogenic genes, including Cyclin D1 and CDC25A [25, 26]. As ROS is known to activate the STAT3 pathway, we next tested the role of GSTP1 overexpression on STAT3 activation and the expression of downstream signaling components. As it is shown in Figure 6(a), overexpression of GSTP1 increased both STAT3 total protein and phosphorylation STAT3. Addition of N‐acetylcysteine (NAC) before hypoxia treatment presented no detectable change in phosphorylation of STAT3, indicates that oxidative stress‐induced ROS is critical in enhancing phosphorylation of STAT3, and overexpressed GSTP1 may stimulate p‐STAT3 via regulating ROS. We then detected downstream targets of STAT3, including Cyclin D1 and CDC25A. As it is shown in Figure 6(b), overexpressed GSTP1 significantly increased both Cyclin D1 and CDC25A protein levels, indicated that overexpressed GSTP1 activates STAT3/Cyclin D1 signaling, which thus regulates malignant behaviors.

Figure 6Overexpression of GSTP1‐stimulated STAT3/Cyclin D1 signaling. (a) After being cultured under normoxia or hypoxia for 24 hours, GSTP1, STAT3, and phosphorylation of STAT3 (p‐STAT3) were detected by performing western blot. *P < 0.05, vs. normoxia/vector group; ^#^ *P* < 0.05, vs. hypoxia group. (b) After GSTP1 overexpression, downstream genes of STAT3, including cyclin D1 and CDC25A were detected by performing western blot. *P < 0.05, vs. normoxia/vector group.

**Figure:** (a)

**Figure:** (b)

## 4. Discussion

In the early gestation period, hypoxia is the typical extrinsic factor regulating trophoblast physiological processes, including cell proliferation, migration, and invasion [5, 6]. In this study, GSTP1 was expressed in trophoblasts of the placenta and trophoblast cells. Compared with full‐term placental tissues, GSTP1 is overexpressed in trophoblast sections in placental tissues of the first trimester, which was further confirmed by western blotting. In our in vitro study, we overexpressed GSTP1 in JEG3, a trophoblast‐like cell line, and found its promoting effects on cell viability, proliferation, colony formation, migration, and invasion. Then, we simulated the physiological hypoxic conditions of early pregnancy by culturing cells in a 3% O_2_ incubator and found that GSPT1 and HIF‐1*α* were obviously stimulated. Overexpression of GSTP1 significantly scavenges ROS, which accumulate after hypoxia exposure. We hypothesized that the expression of GSTP1 in trophoblasts is relevant to physiological hypoxia in early pregnancy. Hypoxia‐induced GSTP1 significantly increased GST activity and thus potentially decreased ROS accumulation. According to our results, we found that trophoblast cell behaviors were promoted by GSTP1, in agreement with previous reports [27–29]. These findings indicate that GSTP1 exerts protective effects on hypoxia by scavenging ROS induced by hypoxia exposure. Considering the importance of trophoblast proliferation and invasion of maternal spiral arterioles during early pregnancy, GSTP1 may play a critical role in preventing PE.

RETRACTED

In vitro studies employing cancer cells showed that GSPT1 exerted promoting effects on malignant behaviors [20, 31]. Wang et al. found that in colorectal cancer cells, overexpression of GSTP1 promotes proliferation, invasion, and metastasis [20]. It has also been reported that in glioblastoma, GSTP1 decreases ROS accumulation and promotes cell proliferation [31]. In our study, as expected, hypoxia exposure stimulated HIF‐1*α* and GSTP1. HIF‐1*α* is a critical transcriptional regulator under hypoxic conditions. In this study, we failed to evaluate whether overexpression of GSTP1 after hypoxia exposure is dependent on transcriptional regulation of HIF‐1*α*, which is worth further investigation.

The present study detected GSTP1 and STAT3 in JEG3 cells after normoxia or hypoxia exposure and found that GSTP1 was positively correlated with the expression of STAT3 and its phosphorylation (p‐STAT3). After hypoxia exposure, GSTP1, STAT3, and p‐STAT3 levels were increased. Notably, the addition of NAC significantly decreased the phosphorylation of STAT3 but did not affect total STAT3, which was stimulated by hypoxia. These results indicate that the upregulation of STAT3 is dependent on GSTP1 and that the increase in p‐STAT3 is dependent on accumulated ROS induced by hypoxia exposure. Briefly, the total amounts of STAT3 and the phosphorylated form of STAT3 were regulated in different manners.

After hypoxia exposure, apoptosis was significantly increased, which was partially reversed by GSTP1 overexpression. This raised the question of whether endogenous GSTP1 induced by hypoxia exposure exerts protective effects on apoptosis. In further investigation, it will be worth employing lentivirus containing shRNA targeting GSTP1 for knockdown, by which the protective effects of endogenous GSTP1 could be further confirmed.

RETRACTED

## 5. Conclusion

Cellular ROS accumulation is subject to tight redox regulation, and disturbance of ROS balance is a critical cause of cellular damage and injury in pregnancy 30. Here, we found that ROS accumulated by hypoxia exposure are markedly scavenged by overexpressed GSTP1, which agrees with the previous finding that GSTP1 contributes to preventing ROS accumulation [22]. GSTP1 is one of the GST family members that catalyze intracellular detoxification reactions by conjugating GSH with hydrophobic and electrophilic compounds [24]. Indeed, upregulated GSTP1 promotes GST activity, which contributes to scavenging accumulated ROS [32]. In addition, because the current study highlights a key role of GSTP1 in regulating ROS levels under hypoxic conditions, it proposes that regulating GSTP1 may be a promising approach to protect against PE.

## Conflicts of Interest

The author(s) declare that they have no conflicts of interest.

## Authors’ Contributions

LJC and CJA designed the experiments. LJC, GLC, and LXG performed experiments on cell sorting and related cellular experiments. LXG and YPW are responsible for data collection and performed statistical analysis. LJC and GLC are considered as co‐first authors. All authors read and approved the final manuscript.

## Data Availability

All data generated or analyzed during this study are included in this published article.
